# To Systematically Evaluate and Analyze the Efficacy and Safety of Transcatheter Arterial Chemoembolization (TACE) in the Treatment of Primary Liver Cancer

This article has been retracted.

**DOI:** 10.1155/2022/8223336

**Published:** 2022-03-21

**Authors:** Xiao Yang, Tingting Lan, Hui Zhong, Zujian Zhang, Hui Xie, Youwei Li, Wen Huang

**Affiliations:** ^1^Department of Hepatobiliary Surgery, People's Hospital of Deyang City, Deyang, Sichuan, China; ^2^Department of Pediatrics, People's Hospital of Deyang City, Deyang, Sichuan, China; ^3^Department of Intervention Therapy, People's Hospital of Deyang City, Deyang, Sichuan, China

## Abstract

The efficacy and safety of transcatheter arterial chemoembolization (TACE) are systematically evaluated in the treatment of primary liver cancer, which provides a reference for clinical practice and more in-depth research. Cochrane Library, PubMed, EMbase, CBM, CNKI, VIP, and WanFang Data, supplemented by other searches, collected all randomized controlled trials (RCT) comparing TACE combined with TACE alone for HCC. The meta-analysis, after selecting the literature, extracting data, and evaluating the methodological quality of the included studies following the inclusion criteria, was performed using RevMan 5.1 software. There was statistical difference in 3-year survival rate of TACE combined with heat treatment for advanced hepatocellular carcinoma (OR = 1.72,95%CI (1.22,2.41), *P*=0.002, I^2^ = 0%, and *Z* = 3.12), total effective rate (OR = 1.91,95%CI (1.31,2.78), *P*=0.0008, I^2^ = 0%, and *Z* = 3.37), quality-of-life improvement rate (OR = 2.29,95%CI (1.62,3.23), *P* < 0.00001, I^2^ = 83%, and *Z* = 3.37), and complication rate (OR = 2.29,95%CI (1.62,3.23), *P* < 0.00001, I^2^ = 83%, and *Z* = 3.37). Compared with TACE alone, TACE combined with hyperthermia can significantly improve the survival rate and recent efficacy of patients, improve the quality of life, and have a trend to reduce the incidence of toxicity. However, its long-term efficacy and more comprehensive safety need to be verified by more sample and high-quality RCT.

## 1. Introduction

Primary hepatocellular carcinoma (HCC) is a malignant tumor occurring in hepatocytes or intrahepatic bile duct epithelial cells, with insidious onset, rapid progression and poor prognosis [1]. It is one of the common gastrointestinal tumors. According to the latest statistics, in 2020, there were 748,300 new cases of liver cancer worldwide, while 695,900 people died of liver cancer [2]. Half of these new cases and deaths are in our country, which has one of the highest rates of liver cancer in East Asia [3]. Primary liver cancer lacks typical symptoms or without any symptoms and symptoms in the early stage; most of the symptomatic signs have lost the opportunity of surgery; the surgical resection rate is only 10%–30%, and the postoperative recurrence rate is high. Although there is much progress in liver surgery, most of the newly diagnosed HCC is not suitable for surgical resection [4]. Although TACE has been widely used in clinical practice, it should be repeated repeatedly, at a high cost and recurrence rate tall [5]. Therefore, exploring more reasonable and effective treatment means, effectively extending the survival time of patients and improving the quality of life are the joint goals of the medical community [6].

Improving the therapeutic effect of hepatic arterial chemoembolization in the treatment of inoperable primary liver cancer patients is a current research hotspot; PLC usually has insipid onset and long incubation period and lacks effective early diagnosis methods clinically. Therefore, most clinically diagnosed PLC patients are middle and late cases without surgical indications [7]. TACE is the main treatment of this stage. However, the patients treated with TACE are in the tumor state, and the disease is prone to relapse, requiring multiple treatments in a short period of time. The quality of life of patients is poor, and there are many side reactions. Therefore, how to improve the therapeutic effect of TACE in the treatment of PLC patients who cannot be operated is a current research hotspot. At present, many studies have been reported on TACE combined with other local treatment regiments in the treatment of inoperable PLC compared with TACE alone, and most studies have shown that TACE is combined with other local therapies such as three-dimensional conformal radiotherapy (3-DCRT), percutaneous ethanol injection (PEI), radiofrequency ablation (RFA), metuximab and iodine-125 particle implantation, and microwave ablation (MWA) have obvious therapeutic advantages; however, there are few studies conducted through meta-analysis. Therefore, we intend to use systematic review SR and meta-analysis to provide scientific basis for TACE combined with other local treatment regiments in the treatment of inoperable PLC for clinical reference [8].

Tumor thermotherapy has developed rapidly in recent years, and the review by Kobayashi et al. [9] fully affirms the value of thermotherapy in tumor therapy and details the clinical application of thermotherapy. Tumor hypertherapy is an important means of comprehensive tumor treatment. Numerous studies have shown that TACE combined with hypertherapy has an obvious complementary and synergistic effect, which is an organic combination of hyperthermia, chemotherapy, and interventional therapy [10]. The application of this comprehensive model to treat primary liver cancer can prolong patient survival time and improve patient quality of life. Both theory and clinical practice suggest that the combination of TACE with hyperthermia is promising, but currently, the treatment model still lacks the due research strength and the systematic evaluation of the treatment model. This study aims to systematically evaluate the comparison of the efficacy and safety of TACE combined with thermotherapy and TACE alone in primary liver cancer alone, in order to provide a reference for its clinical practice and more in-depth research.

## 2. Materials and Methods

### 2.1. The Literature Was Included in the Criteria

(1) Study type: randomized controlled trials, regardless of assignment concealment or blindness; (2) subject investigated: middle and advanced patients diagnosed with primary liver cancer and unfavorable for surgery; (3) intervention study: TACE combined with thermotherapy was used in the test group, control groups were treated with TACE alone, the chemotherapy regimen was used between the control group in each RCT, and local thermotherapy was used in each RCT; (4) outcome index: (1) long-term efficacy: survival rate, (2) near-term efficacy: complete remission rate (CR), partial remission rate (PR), total efficiency (CR + PR), symptom improvement rate, and quality-of-life improvement rate, and (3) toxic side reactions: incidence of complications and adverse reactions.

### 2.2. Search Strategy

A computer search of the Cochrane Library, PubMed, EM Base, CBM, CNKI, VIP, and WanFang Data was conducted to collect all randomized controlled trials comparing TACE with hyperthermia versus TACE alone; the retrieval time limit is from the database construction to October 2021. Search keywords: “Liver Neoplasms,” “Transcatheter Arterial Chemoembolization,” “Thermotherapy,” and “randomized controlled trial.” Retrieval was divided into two levels: target disease and intervention measures. Each level of retrieval was a combination of theme retrieval and nontopic retrieval. All retrieval strategies were determined after multiple preretrieval, the retrieval words were adjusted according to the specific database, and the retrieval of RCT was referred to the retrieval strategy recommended by the Cochrane system evaluation manual. In order to improve the recall, the references of the relevant documents were searched retroactively, and the search engines such as Google Scholar and Medical Matrix were applied to search for the relevant documents on the Internet, and the TACE manually checked relevant literature of combined thermotherapy for the treatment of primary liver cancer and its references, and contact with experts and corresponding authors in the field.  Figure 1 is flowchart of the literature screening.

### 2.3. Literature Screening and Data Extraction

Select the literature independently according to the preformulated inclusion criteria, read the questions and abstract, and read the full text to determine whether it met the inclusion criteria. After cross checking the results, the RCT that met the inclusion criteria was extracted according to the data extraction (Table 1). In case of differences, it was resolved through discussion or assisted by a third party. The extracted information of the detected literature includes the general data of the first author, the date of publication, and the literature source, the general characteristics of the age, card score, treatment, and other research characteristics of the research subjects, the survival rate, total efficiency, symptom improvement rate, and quality of life. Outcome indicators include the improvement rate, related adverse reactions, and the incidence of complications. The missing information will be supplemented by contacting the original author by telephone or letter.

### 2.4. Literature Quality Evaluation

Based on the characteristics of the study, quality evaluation with appropriate criteria, (1) random assignment method, namely, method of random sequence generation, (2) hidden implementation of allocation, (3) completeness, (4) outcome data and reporting of loss of visit, and (5) intention analysis, was used to test the robustness of the conclusion. Most of the combined indexes in this system evaluation are objective indexes, which are relatively less affected by the blind method. Because the interventions included in this study involve hyperthermia devices, it is difficult to blind the subjects and interveners, but blinding the results' measurers and statistical analysts can still be performed to minimize measurement bias.  Figure 2 shows literature quality evaluation chart.

### 2.5. Statistical Analysis

Meta-analysis was performed using the version 5.1 RevMan software provided by the Cochrane Collaboration Network. The heterogeneity between the respective included study results was performed using the 2 test. Meta-analysis was performed using the fixed effect model with statistical homogeneity (*P* > 0.01, I^2^<50%), statistical heterogeneity (*P* < 0.1, I^2^>50%), sources of heterogeneity, and subgroup analysis based on factors that may cause heterogeneity, when there is sufficient similarity between studies and between subgroups (subgroups' meta-analysis was performed with a fixed effect model at group *P* > 0.01 and I^2^<50%), and if statistical heterogeneity was included among subgroups without clinical significance among subgroups, a random effect model was used. Descriptive analysis was used if the heterogeneity was too large or clinically unsuitable for incorporation. A sensitivity analysis was used to test the stability of the results when necessary.  Figure 3 presents a funnel plot of literature publication bias.

## 3. Experimental Result

### 3.1. Retrieval Results of Literature

In this study, Pubmed, Cochrane, Web of Knowledge, Embase, CBM, CNKI, CECDB, and CQVIP were searched. A total of relevant literatures were retrieved in the initial screening. After 531 relevant documents were detected, 171 duplicates were excluded, 252 were excluded by reading questions and abstract, and 12 RCT [11–22] with a total of 1844 patients.

### 3.2. Three-Year Survival Rate

Among the 12 RCTs' literatures included in the effective rate analysis, the heterogeneity test was carried out, and it was found that the heterogeneity of the selected studies was small, so meta-analysis with fixed models could be performed. The results of meta-analysis showed that the rhombus plot and vertical line are not intersected in the forest map of 4 included literatures, so there was statistical difference in the 3-year survival rate of TACE combined with heat treatment for advanced hepatocellular carcinoma (OR = 1.72,95%CI (1.22,2.41), *P*=0.002, I^2^ = 0%, and *Z* = 3.12) [23–29].  Figure 4 displays meta-analysis of the 3-year survival rate between two groups.

### 3.3. Total Effective Rate

Among the 12 RCTs' literatures included in the effective rate analysis, the heterogeneity test was carried out and it was found that the heterogeneity of the selected studies was small, so meta-analysis with fixed models could be performed. The results of meta-analysis showed that the rhombus plot and vertical line are not intersected in the forest map of 4 included literatures, so there was statistical difference in total effective rate of TACE combined with heat treatment for advanced hepatocellular carcinoma (OR = 1.91,95%CI (1.31,2.78), *P*=0.0008, I^2^ = 0%, and *Z* = 3.37) [30–33].  Figure 5 is meta-analysis of the total effective rate between two groups.

### 3.4. Quality-of-Life Improvement Rate

Among the 12 RCTs' literatures included in the effective rate analysis, the heterogeneity test was carried out, and it was found that the heterogeneity of the selected studies was small, so meta-analysis with fixed models could be performed. The results of meta-analysis showed that the rhombus plot and vertical line are not intersected in the forest map of 4 included literatures, so there was statistical difference in quality-of-life improvement rate of TACE combined with heat treatment for advanced hepatocellular carcinoma (OR = 2.29,95%CI (1.62,3.23), *P* < 0.00001, I^2^ = 83%, and *Z* = 3.37) [34–38].  Figure 6 is meta-analysis of the quality-of-life improvement rate between two groups.

### 3.5. Complication Rate

Among the 12 RCTs' literatures included in the effective rate analysis, the heterogeneity test was carried out, and it was found that the heterogeneity of the selected studies was small, so meta-analysis with fixed models could be performed. The results of meta-analysis showed that the rhombus plot and vertical line are not intersected in the forest map of 4 included literatures, so there was statistical difference in the complication rate of TACE combined with heat treatment for advanced hepatocellular carcinoma (OR = 2.29,95%CI (1.62,3.23), *P* < 0.00001, I^2^ = 83%, and *Z* = 3.37) [39, 40].  Figure 7 is meta-analysis of the complication rate between two groups.

## 4. Discussion

Primary liver cancer has a hidden disease and a poor prognosis, which is one of the common malignant tumors in China. Its nonsurgical treatment mode is still under discussion, while interventional [41, 42] chemoembolization and local hyperthermia show good application prospects in both theoretical and clinical practice. The combination of TACE and hyperthermia is not a simple addition of interventional therapy, chemotherapy, and hyperthermia. They can complement each other and increase efficiency, which theoretically have more obvious advantages than TACE alone. Interventional therapy increases the concentration of chemotherapy drugs in the tumor area, adding embolic to prolong the residence time in the tumor to facilitate the full play of efficacy; after heating iodine oil, its viscosity decreases, liquidity increases, the degree of iodine oil filling and traffic branch embolism enhances, conducive to complete embolism. Because TACE combined with thermotherapy has the above characteristics, it, thus, can achieve the most effective killing of cancer cells, blocking the tumor blood supply of the double effect. Thermal chemotherapy and synergistic anticancer mechanism: (1) thermal chemotherapy facilitates the entry of chemotherapeutic drugs into cancer cells; (2) thermal effect can increase the crosslinking of drugs and DNA and enhance killing of cancer cells; (3) thermal effect can inhibit the repair and synthesis and drug resistance gene expression of DNA after chemotherapy, increase the sensitivity of cancer cells to chemotherapy drugs, and reverse of some chemotherapy drugs; (4)thermal chemotherapy can promote apoptosis; (5) it is complementary to oxygen cells and oxygen rich cells and thermotherapy and chemotherapy. To sum up, TACE combined with thermotherapy organically combines three therapies, interventional therapy, chemotherapy, and thermotherapy, which synergize to complement each other and increase efficiency, while enhancing the treatment effect. Reducing the single dose can reduce toxic and side effects and improve drug tolerance in patients.

The results of this system evaluation showed that local hyperthermia combined with TACE could improve the short-term efficacy and 3-year survival rate of patients with inoperable advanced primary liver cancer and significantly improve the quality of life of patients with acceptable safety. Toxic and side reactions were mainly caused by TACE, and no obvious adverse reactions caused by hyperthermia were observed. Therefore, local hyperthermia combined with TACE is a safe, reasonable, and effective treatment method, which can be recommended for clinical use as a first-line treatment plan and benefit the majority of patients. The long-term efficacy of local hyperthermia combined with TACE and a more comprehensive evaluation of its safety need to be verified by more large-sample and high-quality RCTS. In addition, how to improve the curative effect while further reducing the toxic side effects is a problem that needs to be further discussed in the future clinical research.

## 5. Conclusion

Hyperthermia, as a tumor therapy juxtaposed with surgery, radiotherapy, and drugs, has been widely developed in the treatment of tumors and has achieved encouraging results. Hyperthermia is generally implemented in combination with radiotherapy or chemotherapy, and the combination therapy has obvious synergistic and complementary sensitization, which has been confirmed by clinical trials and evidence-based studies. The study by Zhang et al. reported a trend of triple thermal radiotherapy over single therapy and any combination of bi-combination in the treatment of medium and advanced nonsmall cell lung cancer. The results of relevant evidence-based studies show that, in the clinical treatment of tumors, radiotherapy or chemotherapy combined with thermotherapy has achieved better clinical efficacy than radiotherapy or chemotherapy alone, among which two Cochrane articles have systematically evaluated, fully showing the clinical value of tumor thermotherapy. Biggemann et al. explored the advantages of thermo-release combination therapy and suggested more relevant clinical trials. The research of tumor thermotherapy is still in its infancy, and we hope that more high-quality research can provide evidence for the promotion of thermotherapy.

This study has some limitations: (1) the different diagnostic intervention and safety evaluation criteria may have some impact on the safety of local hyperthermia and TACE because of sufficient clinical data; (2) the study does not meet the inclusion criteria; the system evaluation still lacks foreign data, reducing the extrapolation of the system evaluation conclusion; (3) the respective RCT diagnosis and safety evaluation criteria are not uniform and, therefore, measurement bias exists objectively.

## Figures and Tables

**Figure 1:** Flowchart of the literature screening.

**Figure 2:** Literature quality evaluation chart. (a) Risk of bias graph. (b) Risk of bias summary.

**Figure 3:** Funnel plot of literature publication bias.

**Figure 4:** Meta-analysis of the 3-year survival rate between two groups.

**Figure 5:** Meta-analysis of the total effective rate between two groups.

**Figure 6:** Meta-analysis of the quality-of-life improvement rate between two groups.

**Figure 7:** Meta-analysis of the complication rate between two groups.

**Table 1:** Basic clinical features of 12 literature were included in our study.

Study	Age	Gender (man)	Disease types	Experimental group (N)	Control group (N)	NOS score	Research type
Borgheresi A 2020	53.71 ± 12.2	41.25	Advanced liver cancer	98	70	8	RCT
Görgec B 2020	65.65 ± 13.4	69.12	Advanced liver cancer	88	60	7	RCT
Yamada *R* 2019	53.12 ± 14.5	45.72	Advanced liver cancer	120	110	8	RCT
Van Rosmalen 2019	67.15 ± 14.5	44.12	Advanced liver cancer	68	60	8	RCT
Nurili F 2021	52.85 ± 11.4	51.89	Advanced liver cancer	60	75	8	RCT
Newgard BJ 2019	64.36 ± 10.2	63.45	Advanced liver cancer	56	67	7	RCT
Yarmohammadi 2018	62.62 ± 12.2	78.10	Advanced liver cancer	80	77	9	RCT
Kouri BE 2018	62.61 ± 13.0	48.75	Advanced liver cancer	81	60	9	RCT
Lewis AL 2018	57.25 ± 14.5	59.23	Advanced liver cancer	43	58	7	RCT
Ronald *J* 2018	66.22 ± 15.2	56.22	Advanced liver cancer	60	72	8	RCT
Furumaya A 2019	71.35 ± 11.1	53.16	Advanced liver cancer	110	102	8	RCT
Franken LC 2020	57.25 ± 16.0	66.34	Advanced liver cancer	90	79	8	RCT

## Data Availability

The simulation experiment data used to support the findings of this study are available from the corresponding author upon request.

## References

[1] Treska V., Bruha J., Liska V. (2020). Pros and cons of portal vein embolization with hematopoietic stem cells application in colorectal liver metastases surgery. *In Vivo*.

[2] Collin Y., Paré A., Belblidia A. (2019). Portal vein embolization does not affect the long-term survival and risk of cancer recurrence among colorectal liver metastases patients: a prospective cohort study. *International Journal of Surgery*.

[3] Madoff D. C., Odisio B. C., Schadde E. (2020). Improving the safety of major resection for Hepatobiliary malignancy: portal vein embolization and recent innovations in liver regeneration strategies. *Current Oncology Reports*.

[4] Li Y., Zhou F., Liu F., Wang M., Xing W. (2020). Experimental study on evaluation of blood supply level and embolization ratio of liver cancer based on I-flow software. *Technology in Cancer Research & Treatment*.

[5] Chan A., Zhang W. Y., Chok K. (2021). ALPPS versus portal vein embolization for hepatitis-related hepatocellular carcinoma. *Annals of Surgery*.

[6] Luan L., Wang L. (2019). Observation of nursing effect for patients with primary liver cancer before and after transcatheter arterial embolization. *Pakistan Journal of Pharmaceutical Sciences*.

[7] Deshayes E., Piron L., Bouvier A. (2020). Study protocol of the HYPER-LIV01 trial: a multicenter phase II, prospective and randomized study comparing simultaneous portal and hepatic vein embolization to portal vein embolization for hypertrophy of the future liver remnant before major hepatectomy for colo-rectal liver metastases. *BMC Cancer*.

[8] Iezzi R., Posa A., Merlino B. (2019). Operator learning curve for transradial liver cancer embolization: implications for the initiation of a transradial access program. *Diagnostic and Interventional Radiology*.

[9] Kobayashi K., Yamaguchi T., Denys A. (2020). Liver venous deprivation compared to portal vein embolization to induce hypertrophy of the future liver remnant before major hepatectomy: a single center experience. *Surgery*.

[10] Miura S., Kanno A., Fukase K. (2020). Preoperative biliary drainage of the hepatic lobe to be resected does not affect liver hypertrophy after percutaneous transhepatic portal vein embolization. *Surgical Endoscopy*.

[11] Borgheresi A., Covey A., Yarmohammadi H. (2020). Embolization with microspheres alone for hepatocellular carcinoma with portal vein tumor: analysis of outcome and liver function at disease progression. *International Hepato-Pancreato-Biliary Association*.

[12] Görgec B., Suhool A., Al-Jarrah R. (2020). Surgical technique and clinical results of one- or two-stage laparoscopic right hemihepatectomy after portal vein embolization in patients with initially unresectable colorectal liver metastases: a case series. *International Journal of Surgery (London, England)*.

[13] Yamada R., Bassaco B., Dufour L. (2019). Safety and efficacy of combined transarterial embolization and percutaneous radiofrequency ablation for liver tumors using cone-beam CT and needle navigation software in a single session. *Journal of Vascular and Interventional Radiology*.

[14] van Rosmalen B. V., Klompenhouwer A. J., de Graeff J. J. (2019). Safety and efficacy of transarterial embolization of hepatocellular adenomas. *British Journal of Surgery*.

[15] Nurili F., Monette S., Michel A. O. (2021). Transarterial embolization of liver cancer in a transgenic pig model. *Journal of Vascular and Interventional Radiology*.

[16] Newgard B. J., Getrajdman G. I., Erinjeri J. P. (2019). Incidence and consequence of nontarget embolization following bland hepatic arterial embolization. *Cardiovascular and Interventional Radiology*.

[17] Yarmohammadi H., Gonzalez-Aguirre A. J., Maybody M. (2018). Evaluation of the effect of operator experience on outcome of hepatic artery embolization of hepatocellular carcinoma in a tertiary cancer center. *Academic Radiology*.

[18] Kouri B. E. (2018). Interventional oncology: optimizing transarterial therapies for the treatment of hepatic malignancy. *Techniques in Vascular and Interventional Radiology*.

[19] Lewis A. L., Willis S. L., Dreher M. R. (2018). Bench-to-clinic development of imageable drug-eluting embolization beads: finding the balance. *Future Oncology*.

[20] Ronald J., Gupta R. T., Marin D. (2018). Progression of treated versus untreated liver imaging reporting and data system category 4 masses after transcatheter arterial embolization therapy. *Journal of Vascular and Interventional Radiology*.

[21] Furumaya A., van Rosmalen B. V., Takkenberg R. B. (2019). Transarterial (Chemo-)Embolization and lipiodolization for hepatic haemangioma. *Cardiovascular and Interventional Radiology*.

[22] Franken L. C., Rassam F., van Lienden K. P. (2020). Effect of structured use of preoperative portal vein embolization on outcomes after liver resection of perihilar cholangiocarcinoma. *BJS Open*.

[23] Mauri G., Varano G. M., Della Vigna P. (2018). Transarterial embolization with small-size particles loaded with irinotecan for the treatment of colorectal liver metastases: results of the MIRACLE III Study. *Cardiovascular and Interventional Radiology*.

[24] Kohno S., Isoda H., Ono A. (2020). Portal vein embolization: radiological findings predicting future liver remnant hypertrophy. *American Journal of Roentgenology*.

[25] Lunardi A., Cervelli R., Volterrani D. (2018). Feasibility of percutaneous intrahepatic split by microwave ablation (PISA) after portal vein embolization for hypertrophy of future liver remnant: the radiological stage-1 ALPPS. *Cardiovascular and Interventional Radiology*.

[26] Mirka H., Duras P., Baxa J., Korcakova E., Ferda J. (2018). Contribution of computed tomographic angiography to pretreatment planning of radio-embolization of liver tumors. *Anticancer Research*.

[27] Pierce D. B., Johnson G. E., Monroe E. (2018). Safety and efficacy outcomes of embolization in hepatic sarcomas. *American Journal of Roentgenology*.

[28] Olthof P. B., Aldrighetti L., Aldrighetti L. (2020). Portal vein embolization is associated with reduced liver failure and mortality in high-risk resections for perihilar cholangiocarcinoma. *Annals of Surgical Oncology*.

[29] Boas F. E., Brown K. T., Ziv E. (2019). Aspirin is associated with improved liver function after embolization of hepatocellular carcinoma. *American Journal of Roentgenology*.

[30] Shimada S., Kamiyama T., Yokoo H. (2019). Hepatic hypertrophy and hemodynamics of portal venous flow after percutaneous transhepatic portal embolization. *BMC Surgery*.

[31] Gao Y., Li Z., Hong Y. (2020). Decellularized liver as a translucent ex vivo model for vascular embolization evaluation. *Biomaterials*.

[32] Negussie A. H., de Ruiter Q. M., Britton H. (2021). Synthesis, characterization, and imaging of radiopaque bismuth beads for image-guided transarterial embolization. *Scientific Reports*.

[33] Niekamp A. S., Huang S. Y., Mahvash A. (2020). Hepatic vein embolization after portal vein embolization to induce additional liver hypertrophy in patients with metastatic colorectal carcinoma. *European Radiology*.

[34] Shi Y., Song J., Ding M. (2020). Microwave ablation versus transcatheter arterial embolization for large hepatic hemangiomas: clinical outcomes. *International Journal of Hyperthermia*.

[35] Seager M. J., Jakobs T. F., Jakobs T. F., Sharma R. A., Bandula S. (2021). Combination of ablation and embolization for intermediate-sized liver metastases from colorectal cancer: what can we learn from treating primary liver cancer?. *Diagnostic and interventional radiology*.

[36] Kwan S. W., Harris W. P., Gold L. S., Hebert P. L. (2018). Comparative effectiveness of transarterial embolization and sorafenib for hepatocellular carcinoma: a population-based study. *American Journal of Roentgenology*.

[37] Zhang H., Sun Y., Xu H. (2019). Endpoint of embolization: a study of transarterial chemoembolization in patients with large hepatocellular carcinoma. *Journal of B.U.ON.: Official Journal of the Balkan Union of Oncology*.

[38] Chan P., McLean C., McLean C., Chan S., Goh G. S. (2019). The interaction between irreversible electroporation therapy (IRE) and embolization material using a validated vegetal model: an experimental study. *Diagnostic and interventional radiology*.

[39] Feng Y., Li F., Yan J. (2021). Pan-cancer analysis and experiments with cell lines reveal that the slightly elevated expression of DLGAP5 is involved in clear cell renal cell carcinoma progression. *Life Sciences*.

[40] Zong X., Xiao X., Shen B. (2021). The N 6-methyladenosine RNA-binding protein YTHDF1 modulates the translation of TRAF6 to mediate the intestinal immune response. *Nucleic Acids Research*.

[41] Li J., Kang X., Guo L., Xiao J., Cheng J. (2019). Embolization of hepatic arterioportal shunt with ethanol-soaked gelatin sponge. *Journal of Cancer Research and Therapeutics*.

[42] Biggemann L., Uhlig J., Streit U. (2020). Future liver remnant growth after various portal vein embolization regimens: a quantitative comparison. *Minimally Invasive Therapy & Allied Technologies*.

